# Three-Dimensional Echocardiography and Coagulation Function Detection in the Prognosis Evaluation of Patients with Acute Myocardial Infarction

**DOI:** 10.1155/2022/5197871

**Published:** 2022-05-28

**Authors:** Yatong Zhang, Zinan Zhao, Li Zheng, Tian Zhang, Xuelin Sun

**Affiliations:** ^1^Department of Pharmacy, Beijing Hospital, National Center of Gerontology, Institute of Geriatric Medicine, Chinese Academy of Medical Sciences, Beijing Key Laboratory of Assessment of Clinical Drugs Risk and Individual Application (Beijing Hospital), Beijing 100730, China; ^2^Department of Pharmacy, China Aerospace Science & Industry Corporation 731 Hospital, Beijing 100000, China

## Abstract

This research was aimed at discussing the application value of coagulation function detection and three-dimensional echocardiography in the prognosis evaluation of acute myocardial infarction (AMI) patients. 72 patients with AMI were divided into the recovered group (good recovery) and unrecovered group (poor recovery) according to the results of postoperative ultrasonography. The left ventricular parameters of the patients were detected by three-dimensional ultrasound, and the coagulation function was also detected. The results showed that 3 months after surgery, the regional end-systolic volume (rESV) and regional end-diastolic volume (rEDV) of the left ventricle in the patients were smaller than the measured values 1 week after surgery. The left ventricular regional ejection fraction (rEF) was greater than the value measured 1 week after surgery, and all the differences were statistically significant (*P* < 0.05). For the end-systolic volume (ESV), end-diastolic volume (EDV), and ejection fraction (EF) (%), the two-dimensional ultrasound results were significantly lower than the three-dimensional ultrasound results, and there were significant differences (*P* < 0.05). Tmsvle6-Dif% of the recovered patients was 14.99 ± 9.88 and 14.37 ± 9.78 3 months and 6 months after surgery, respectively. These were smaller than 30.91 ± 18.63 and 33.51 ± 17.96 of the unrecovered patients; the differences were of statistical significance (*P* < 0.05). Tmsvl6-SD% of recovered patients was 3.69 ± 2.47 and 3.61 ± 1.83 3 months and 6 months after surgery, respectively, which were also smaller than 7.38 ± 4.06 and 7.96 ± 2.82 of unrecovered patients, showing statistically significant difference (*P* < 0.05). The postoperative Tmsvle6-Dif% and Tmsvl6-SD% of the recovered group were lower than those of the unrecovered patients, with the statistically significant differences (*P* < 0.05). The level of coagulation factors in the recovered group was also significantly lower than that in the unrecovered group with the difference statistically significant (*P* < 0.05). The results suggested that three-dimensional echocardiography played an important role in the evaluation of cardiac conditions in AMI patients. The level of coagulation factors varied with the AMI condition of patients, and there was an obvious relationship between them, which could provide a reference value for the prognosis evaluation of patients.

## 1. Introduction

In recent years, the prevalence of acute myocardial infarction (AMI) has been gradually rising. AMI is the myocardial necrosis caused by acute myocardial ischemia, and it is mainly on the grounds of coronary artery diseases [1]. The clinical features include persistent and severe retrosternal pain, elevated serum myocardial enzymes and white blood cell counts, fever, arrhythmia, progressive electrocardiographic changes, heart failure, and even shock [2]. The pathophysiological manifestations are some hemodynamic changes in left ventricular systolic and diastolic dysfunction, such as increased left ventricular end-diastolic pressure, uncoordinated myocardial contraction, and increased end-systolic volume (ESV) as well as end-diastolic volume (EDV). Its severity mainly depends on the infarcted location, duration, and extent of lesions [3]. In AMI, ischemia occurs in the myocardium that supplies blood to the relevant blood vessels at the infarcted location, resulting in abnormal changes in focal systolic function. Therefore, with the comparative analysis of changes in the entire cardiac function, the detection of regional ventricular wall motion can be effectively improved to explore the sensitivity of ventricular systolic dysfunction in patients with AMI [4].

Conventional two-dimensional echocardiography can analyze the changes of overall cardiac function merely, and it generally observes ventricular wall motion with the naked eyes. In addition, it cannot quantitatively analyze ventricular wall motion, and the analyzed slices get certain limitations so that it cannot display the endocardial surface of the left ventricle completely. Thus, its accuracy being questioned [5]. Cardiac magnetic resonance imaging (CMRI) has high temporal and spatial resolution, and it can analyze the volume of cardiac chambers without relying on geometrical shape assumptions. It can directly calculate the shape, size, and volume of cardiac chambers and will not affect its accuracy. It is recognized as the gold standard for measuring cardiac chamber volume and ejection fraction (EF) currently. However, in the measurement of left ventricular volume, the basal plane of the left ventricle needs to be determined manually, and there are subjective factors of the analyst. CMRI examination goes with contraindications or relative contraindications. The examination requires the patients to hold their breath for a long time; for patients who cannot cooperate with the examination, CMRI examination cannot be performed. CMRI is expensive and takes a long time; it is difficult to make a follow-up reexamination [6].

The real-time three-dimensional echocardiography does not rely on the assumption of geometric shape as well. Even in the evaluation of cardiac function under pathological conditions of ventricular deformation and abnormal ventricular wall segmental motion, it can also make an intuitive and accurate quantitative evaluation [7]. Thus, the three-dimensional echocardiography plays a very important role in the diagnosis, efficacy evaluation, and prognosis of patients with heart diseases [8]. It measures cardiac function as the ventricular long-axis end-diastolic image and end-systolic image are selected. It cuts the heart base to the apex into numerous short-axis sections in parallel and depicts the contours and areas of the cardiac chambers and heart wall, respectively. These short-axis sections are accumulated by the computer to accurately estimate the volume of the heart chambers and the weight of the ventricular walls. Therefore, it can accurately, effectively, and quantitatively evaluate the changes of left ventricular configuration and myocardial segment function in AMI patients, and more detailed left ventricular work done information can be provided by three-dimensional echocardiography [9].

Existing studies believe that the incidence and development of AMI are closely related to coronary atherosclerosis, atherosclerotic plaque rupture, and platelet aggregation in the blood to form thrombus on the ruptured plaque surface [10]. Medical works in recent years have shown that abnormal coagulation factors play a very important role in the incidence and pathological mechanism of atherosclerotic cardiovascular diseases. Abnormal coagulation mechanism can lead to increased blood coagulation, which is one of the major causes of coronary thrombosis. Some coagulation factors, such as the factor II (FII), the factor VII (FVII), the factor VIII (FVIII), fibrinogen (Fg), and von Willebrand factor (vWF), are in a close relation to the incidence and development of thrombosis and coronary heart diseases [11]. But so far, there are few reports on the role of coagulation mechanism in the prognosis of AMI surgery.

Therefore, patients with AMI the first time who underwent surgical treatment were chosen. The blood coagulation function test was performed after surgery, and the follow-up echocardiography was made 1 week, 3 months, and 6 months after surgery, respectively. The postoperative recovery of patients was evaluated by three-dimensional ultrasound. The results of traditional two-dimensional ultrasound were compared to explore the possible role of coagulation factors and the application value of three-dimensional ultrasonography in the prognosis of AMI surgery. Thereby, it could provide the data support for clinical improvement of the treatment effect of AMI in the future.

## 2. Research Methods

### 2.1. Research Objects

A total of 72 patients with AMI the first time in hospital from June 2019 to June 2021 were selected, including 39 males and 33 females. The patients were aged 28-79 years old, with an average of (56.27 ± 9.88) years old. All the patients received percutaneous coronary intervention, which was the gold standard that the patients were confirmed with AMI. Their electrocardiogram showed the sinus rhythm. According to the results of postoperative ultrasound examination, they were divided into the recovered group with good recovery, and the unrecovered group with poor recovery. The patients included signed the informed consent, and this research had been approved by ethics committee of hospital.

The included patients met the following inclusion criteria. Their chest pain lasted more than 30 minutes, with characteristic electrocardiographic changes. The enzymatic indicators, myocardial zymogram and troponin, increased. The emergency echocardiography suggested abnormality of segmental wall motion. The patients could be followed up on time and in cooperation with examinations.

The exclusion criteria were as follows: the age of patients > 80 years old. Patients had a history of AMI, or patients were complicated with heart diseases for other causes. Patients suffered from angina pectoris, acute pulmonary embolism, acute pericarditis, etc., which were easily misdiagnosed as AMI. Patients with AMI due to noncoronary atherosclerosis were excluded.

### 2.2. Echocardiography Examination

For the two-dimensional echocardiography, the S5-1 probe was used to probe into the various conventional planes of the heart. The parasternal left ventricular long-axis plane, aortal short-axis plane, mitral valves, short-axis plane of papillary muscle and apex, and apical four-chamber and two-chamber plane were included. The left ventricular end-systolic volume, left ventricular diastolic volume, and left ventricular ejection fraction were analyzed by the two-dimensional Simpson method.

The real-time X5-1 probe was used for the three-dimensional echocardiography. The probe was placed at the apex of the heart, and the direction of the sound beam of the probe was carefully adjusted in the orientation of the apical four-chamber plane until an ideal left ventricular image was obtained. The patients were instructed to hold the breath. The full volume imaging mode was turned on, and the stereo images of four adjacent 15° × 60° narrow-angle pieces were collected through triggering the electrocardiography. The three-dimensional database of 60° × 60° wide-angle pyramid-like full volume imaging was then formed. The images were stored on the hard disk for offline analysis.

The images of the two echocardiographies above were all acquired by the same experienced physician.

### 2.3. Ultrasound Image Analysis

Qlab (8.1) quantitative analysis software was applied to analyze the three-dimensional data. The sagittal and coronal planes were adjusted to be in the middle of the left ventricle at end-diastole and end-systole, and the transverse plane was at the level of the mitral valve annulus. Then, 5 left ventricular endometrial sampling points were selected, namely, the septum and lateral wall sampling points at the level of the mitral valve annulus in the four-chamber view, the anterior and inferior wall sampling points at the level of the mitral valve annulus in the two-chamber view, and the apical sampling point of the four-chamber view or two-chamber view. The instrument drew the dynamic three-dimensional endocardial contour immediately and automatically. If the endocardium depicted by the instrument was not in good agreement with the actual situation, local adjustments could be made manually frame by frame to achieve the best match. The sequence analysis function key was started, and the system would calculate and display the overall and segmental volume-time curves of the left ventricle automatically. The standard deviation (SD) and the maximum difference (Dif) of the time to minimal systolic volume (Tmsv) from the left ventricular 16th segment and their percentage of the cardiac cycle (Tmsvle6-SD, Tmsvl6-SD%, Tmsvl6-Dif, and Tmsvl6-Dif%) were also calculated automatically. The left ventricle was divided into 17 segments, which were displayed with bull's eye diagram and volumetric shell image in 17 different colors. The analysis software could automatically export a data table, as the volume value of each point and the time interval from the point to the start point of the *O*-wave of the electrocardiogram were included. With the table, the regional end-diastolic volume (rEDV) and regional end-systolic volume (rESV) of each segment of the left ventricular wall were calculated. The regional ejection fraction (rEF) could be calculated for rEF = [(rEDV − rESV)/rEDV] × l00% [12].

Three-dimensional echocardiography was performed 1 week, 3 months, and 6 months, respectively, after surgery, and the above indicators were measured and calculated repeatedly.

### 2.4. Detection Methods of Blood Function

For the collection, the patients in both groups were sampled with peripheral venous blood within 2 hours of admission. None of heparin, low molecular weight heparin, bivalirudin, and other anticoagulant drugs were used before blood collection. The anticoagulation treatment was done with 3.8% sodium citrate at a ratio of 1 : 9. The samples were centrifuged within 1 hour at normal room temperature (3000 rpm for 15 minutes). Then, the upper plasma was taken and stored in a -80°C refrigerator for the detection of coagulation factors FII, FVII, FVIII, Fg, and vWF.

For the detection, the levels of FII, FVII, FVII, Fg, and vWF in the plasma of the research objects were detected by the enzyme-linked immunosorbent double monocloned antibody method. The detection of all coagulation factors should be completed within 3 months after the plasma was stored.

### 2.5. Statistical Methods

SPSS17.0 was used, and the continuous variable data were represented as mean ± standard deviation ($\bar{x}\pm s$). All data were tested for normal distribution and homogeneity of variance. The comparison of parameters between two groups was performed by independent sample test. A difference was considered to be statistically significant as *P* < 0.05.

## 3. Research Results

### 3.1. Parameters of Various Segments of AMI Patients after Treatment

The detection results were shown in Figures 1–6, in which it was displayed with the changes in functional parameters of each segment of patients during the postoperative follow-ups. 3 months after surgery, the rESV and rEDV of the infarcted segment and the peripheral area were smaller than the values measured 1 week after surgery, while rEF became greater, and the differences were statistically significant for *P* < 0.05. 6 months after surgery, for the infarcted segment and the peripheral area, rESV and rEDV were smaller than those 3 months after surgery, and rEF was greater than that 3 months after surgery, but the differences were not statistically significant as *P* > 0.05.

### 3.2. Comparison of Left Ventricular EDV, ESV, and EF Measured by Different Methods

The EDV, ESV, and EF (%) of two-dimensional echocardiography were 99.28 ± 19.42, 53.21 ± 10.31, and 47.58 ± 4.21, respectively. Those of the real-time three-dimensional echocardiography were 110.76 ± 19.59, 68.46 ± 9.88, and 37.94 ± 5.03, respectively. As shown in Figure 7, there was a significant difference in each item between the two methods, *P* < 0.05.

### 3.3. Comparison of the Left Ventricular Parameters in the Overall Systole and the Synchronization of Ventricular Wall Motion

Tmsvle6-Dif% of the recovered patients was 14.99 ± 9.88 and 14.37 ± 9.78 3 months and 6 months after the surgery, respectively. These were smaller than the 30.91 ± 18.63 and 33.51 ± 17.96 of the unrecovered patients, and the differences were statistically significant for *P* < 0.05. Tmsvl6-SD% of the recovered patients was 3.69 ± 2.47 and 3.61 ± 1.83, respectively, 3 months and 6 months after surgery, smaller than 7.38 ± 4.06 and 7.96 ± 2.82 of unrecovered patients, suggesting that the differences were of statistical significance for *P* < 0.05. The details were represented in Figure 8 below.

### 3.4. Comparison of Coagulation Factors between the Two Groups

The levels of coagulation factors FII, FVII, FVIII, Fg, and vWF in the recovered group were 48.22 ± 7.85 *μ*g/L, 204.93 ± 9 ng/mL, 6.6 ± 3.5 nmol/L, 234.5 ± 8.7 U/L, and 166.9 ± 2.8 pg/mL, respectively. The levels of these coagulation factors in the unrecovered group were 78.12 ± 9.03 *μ*g/L, 241.18 ± 10 ng/mL, 16.3 ± 4.6 nmol/L, 266.4 ± 9.2 U/L, and 180.5 ± 3.3 pg/mL, respectively. It was found from the comparative results between the two groups that the levels of coagulation factors in the recovered group were lower than those in the unrecovered group, with the differences statistically significant as *P* < 0.05 (Figure 9).

## 4. Discussion

Studies have shown that left ventricular EF is related to the prognosis of AMI, and it is an important indicator to measure the systolic function of patients with heart failure [13]. It has been confirmed that the morphology of the left ventricle evolves from ellipsoid-like to be spherical after AMI, and the morphological changes of the left ventricle are closely related to cardiac function [14]. The prognosis of the treatment was mainly evaluated according to the left ventricular conditions after surgery of the patients. The results showed that 3 months after surgery, the rESV and rEDV of the infarcted segment as well as the peripheral area were smaller than those 1 week after the surgery, but rEF was greater; the differences got the statistical significance due to *P* < 0.05. rESV and rEDV 6 months after surgery were smaller than the measured values 3 months after the surgery, and rEF was greater as well, but the differences were not statistically significant at all as *P* > 0.05. This indicated that the patients' condition improved significantly after surgery, but perhaps because of the small sample size, there were changes but no significant difference 6 months after surgery.

In reality, echocardiography is commonly used to evaluate cardiac function, and *M*-mode and two-dimensional echocardiography techniques are commonly used for cardiac function evaluation in clinical work. The cardiac cavity becomes irregular in the morphology, which deviates from the assumed model; so, there will be a relatively large error [15]. However, real-time three-dimensional echocardiography is not limited by any geometric assumption, and the three-dimensional spatial structure of the heart can be quickly displayed. The observation indicators can also be accurately detected in three-dimensional space by relying on the realistic geometric shape of the ventricle [16]. After comparative analysis, the EDV, ESV, and EF (%) of two-dimensional echocardiography were measured to be 99.28 ± 19.42, 53.21 ± 10.31, and 47.58 ± 4.2, respectively. The results of real-time three-dimensional echocardiography were 110.76 ± 19.59, 68.46 ± 9.88, and 37.94 ± 5.03, respectively; there were the significant differences between the two groups with *P* < 0.05. Such results were considered to be due to the existence of abnormal left ventricular wall motion and ventricular remodeling. When the volume of the left ventricle was obtained as the apical two-chamber and four-chamber views were monitored, segments with abnormal wall motion were not included. This resulted in the left ventricular volume that was underestimated by two-dimensional echocardiography, while the 17-segment method used to measure the left ventricular volume in three-dimensional echocardiography included all segments with normal and abnormal wall motion. Thus, the three-dimensional echocardiography can truly reflect the changes in left ventricular volume and calculate EF accurately [17]. Therefore, for AMI patients, the measurement by the two-dimensional Simpson method was inaccurate due to the existence of ventricular deformation and abnormal ventricular wall motion, while the results obtained by the real-time three-dimensional echocardiography were more accurate.

Researches have shown that after AMI, the left ventricle changes from the overall, rapid, and synchronous, spherical-like ventricular systole to slow, asynchronous, segmental ventricular wall systole. With the exacerbation of the degree of myocardial ischemia and the incidence of myocardial necrosis, once the segments of ventricular muscle cannot coordinately contract in a certain order, it is difficult to generate effective pressure. This will affect the pumping function of the heart; that is, the asynchronous motion of the heart is closely related to the degree of deterioration of cardiac function [18]. It was suggested that the Tmsvle6-Dif% of recovered patients 3 months and 6 months after surgery was 14.99 ± 9.88 and 14.37 ± 9.78, respectively. These were lower than those of unrecovered patients with the value of 30.91 ± 18.63 and 33.51 ± 17.96, having the statistical significance in the differences for *P* < 0.05. The Tmsvl6-SD% of the recovered patients was 3.69 ± 2.47 and 3.61 ± 1.83, respectively, 3 months and 6 months after the surgery. Compared with 7.38 ± 4.06 and 7.96 ± 2.82 for the unrecovered patients, these results were relatively lower, and the differences were statistically significant for *P* < 0.05. It was indicated that the patients in the recovered group had less damage to left ventricular function and recovered to a certain extent. The values of Tmsvle6-Dif% and Tmsvl6-SD% gradually decreased, and the prognosis of these patients was better. Some studies have shown that the synchronization parameters of ventricular wall motion can be utilized as important parameters for evaluating the prognosis of AMI patients. The real-time three-dimensional echocardiography time-volume curve can automatically analyze the parameters of wall-motion synchronization parameters (Tmsvl6-Dif%, Tmsvl6-SD%, etc.), and the method is simple and accurate [19].

The results of this work suggested that the levels of coagulation factors FII, FVII, FVII, Fg, and vWF in the recovered group were detected to be 48.22 ± 7.85 *μ*g/L, 204.93 ± 9 ng/mL, 6.6 ± 3.5 nmol/L, 234.5 ± 8.7 U/L, and 166.9 ± 2.8 pg/mL, respectively. Those of the unrecovered group were detected as 78.12 ± 9.03 *μ*g/L, 241.18 ± 10 ng/mL, 16.3 ± 4.6 nmol/L, 266.4 ± 9.2 U/L, and 180.5 ± 3.3 pg/mL, respectively. With the comparison between the two groups, the levels of coagulation factors in the recovered group were lower than those in the unrecovered group, showing the statistically significant differences with *P* < 0.05. It proved that the increase of coagulation factor levels was related to the development of AMI, and it had a reference value in the evaluation of the prognosis of AMI patients. A large number of studies have demonstrated that coagulation factors play a vital role in the occurrence and development of cardiovascular diseases. Ding et al. (2020) [20] found that the levels of coagulation factors in patients were significantly downregulated after treatment.

## 5. Conclusion

The changes of coagulation function were detected in patients with AMI after treatment, and three-dimensional echocardiography was applied to detect left ventricular parameters. The results suggested that real-time three-dimensional echocardiography could more accurately evaluate the cardiac function and left ventricular volume changes of patients. It could also help doctors evaluate the location of the infarcted segment effectively. It was of great significance for the clinical treatment and prognosis of AMI patients, reduction of the mortality, and improvement of the prognosis, having an application value. The levels of coagulation factors changed with the condition of AMI patients, which could provide reference for the prognosis evaluation of patients, and were worthy of promotion. However, due to limited conditions, the included sample size was small, and there might be certain deviations in the specific data results; thus, further research was required in the future.

## Figures and Tables

**Figure 1:** Analysis of the systolic function of the basal segment of the anterior septum and the anterior wall. ^∗^Compared with the results 7 weeks after surgery, *P* < 0.05.

**Figure 2:** Analysis of the systolic function of the middle segment of the anterior septum and wall. ^∗^Compared with those 7 weeks after surgery, *P* < 0.05.

**Figure 3:** The systolic function of the apical segment of the anterior wall and septum. ^∗^Compared with the corresponding value 7 weeks after surgery, *P* < 0.05.

**Figure 4:** The systolic function of the basal segment of the posterior and inferior walls. ^∗^Compared with the data 7 weeks after surgery, *P* < 0.05.

**Figure 5:** Comparison of the systolic function of the middle segment of the posterior and inferior walls. ^∗^Compared with those 7 weeks after surgery, *P* < 0.05.

**Figure 6:** Comparison of the systolic function of the apical segment of the inferior and posterior walls. ^∗^Compared with the corresponding results 7 weeks after surgery, *P* < 0.05.

**Figure 7:** Comparison of left ventricular EDV, ESV, and EF between the different methods. ^∗^Compared with the results measured by two-dimensional echocardiography, *P* < 0.05.

**Figure 8:** The parameters of the overall systole and ventricular wall motion synchronization of the left ventricle. ^∗^Compared with the results of recovered group, *P* < 0.05.

**Figure 9:** Levels of coagulation factors in plasma between the two groups. ^∗^Compared with the unrecovered group, *P* < 0.05.

## Data Availability

The data used to support the findings of this study are available from the corresponding author upon request.
